# A Multistrategy-Integrated Learning Sparrow Search Algorithm and Optimization of Engineering Problems

**DOI:** 10.1155/2022/2475460

**Published:** 2022-02-23

**Authors:** Zikai Wang, Xueyu Huang, Donglin Zhu

**Affiliations:** School of Information Engineering, Jiangxi University of Science and Technology, Ganzhou, Jiangxi 341000, China

## Abstract

The swarm intelligence algorithm is a new technology proposed by researchers inspired by the biological behavior of nature, which has been practically applied in various fields. As a kind of swarm intelligence algorithm, the newly proposed sparrow search algorithm has attracted extensive attention due to its strong optimization ability. Aiming at the problem that it is easy to fall into local optimum, this paper proposes an improved sparrow search algorithm (IHSSA) that combines infinitely folded iterative chaotic mapping (ICMIC) and hybrid reverse learning strategy. In the population initialization stage, the improved ICMIC strategy is combined to increase the distribution breadth of the population and improve the quality of the initial solution. In the finder update stage, a reverse learning strategy based on the lens imaging principle is utilized to update the group of discoverers with high fitness, while the generalized reverse learning strategy is used to update the current global worst solution in the joiner update stage. To balance exploration and exploitation capabilities, crossover strategy is joined to update scout positions. 14 common test functions are selected for experiments, and the Wilcoxon rank sum test method is achieved to verify the effect of the algorithm, which proves that IHSSA has higher accuracy and better convergence performance to obtain solutions than 9 algorithms such as WOA, GWO, PSO, TLBO, and SSA variants. Finally, the IHSSA algorithm is applied to three constrained engineering optimization problems, and satisfactory results are held, which proves the effectiveness and feasibility of the improved algorithm.

## 1. Introduction

In recent years, new intelligent optimization algorithms have emerged continuously and have been practically applied in medical treatment [1, 2], finance [3], production scheduling [4], and other fields. Besides, it has been proved to be remarkably effective. Since the end of the last century, scholars from all over the world have been inspired by social behavior [5], trying to simulate the behavior characteristics of biological populations in nature, and proposed algorithms such as Ant Colony Algorithm (ACO) [6, 7], Particle Swarm Optimization (PSO) [8, 9], Whale Optimization Algorithm (WOA) [10], Grey Wolf Optimization Algorithm (GWO) [11], and a series of swarm intelligence optimization algorithms. Most of the modeling process of these algorithms is based on the characteristics of the biological population, such as foraging [12], reproduction [13], and hunting [14], which vividly simulate the main behaviors in social actions. In 2020, Xue J and Shen B jointly proposed the Sparrow Search Algorithm (SSA) [1] based on the foraging behavior and backfeeding behavior of sparrow populations. The formula and control parameters of algorithm are not complex and are easier to be understood and implemented relatively. Experiments show that SSA's optimization capability is stronger than the particle swarm optimization algorithm proposed in 1995 and the grey wolf algorithm proposed in 2014, with better convergence accuracy, faster convergence speed, and better stability. However, compared with the existing swarm intelligence optimization algorithm, the SSA also has certain shortcomings, such as longer running time, and a greater possibility to fall into a local optimal solution due to the excessively fast convergence speed, so that the global optimization ability is insufficient.

In order to strengthen the optimization effect of the algorithm and balance the capabilities of exploration and mining, researchers have proposed a series of improved methods for the original sparrow search algorithm model to improve the problem of easily trapping into local optimality. Of course, these improved methods of the swarm intelligence optimization algorithm have been used in various research fields, and the application has been realized extensively. Lv et al. [2] introduced a chaotic sequence to chaotically perturb some individuals, which fell into the local optimum, in order for the SSA to be jumped out of the restriction and continue to search for the global optimum solution. At the same time, the integrated Cauchy-Gaussian mutation operator is combined together to avoid the stagnation of optimization by changing the position of the elite sparrow in the search space. Zhu [15] introduced an adaptive learning factor to solve the problem that the convergence trend will slow down and the convergence accuracy will be reduced under a limited number of iterations, which are the shortcomings of the SSA. At the same time, the ASSA is applied to the optimization and identification of PEMFC stack parameters. Mao and Zhang [16] fused the sine cosine algorithm and the Levy flight strategy on the basic SSA, performed disturbance mutation at the optimal solution position, which enhanced the ability of the algorithm to escape locally, and greatly increased the accuracy of the solution. Liu et al. [17] and others introduced an improved sparrow search strategy to apply to the route planning problem of UAVs, which solved the inefficiency of path planning in the complex three-dimensional flight process. Yuan et al. [18] utilized the center of gravity reverse learning mechanism to initialize the population, which made the population distribution wider. A learning factor is put forward in the update part of the discoverer, and the mutation operator is introduced to increase the mutation processing and reduce the probability of the algorithm falling into the local optimum. Applying it to Distributed Maximum Power Point Tracking (DMPPT) provides conditions for the stable operation of the microgrid. Liu et al. [19] came up with a balanced sparrow search algorithm (BSSA), and the random walk strategy of Levy flight method was exerted to appropriately adjust the local search, which brought the improving efficiency of CNN focus. Besides, they applied it to the medical field to improve MRI image diagnosis of the brain robustness and accuracy of tumors. In order to solve the problem of labeled data classification, Zhang et al. [20] adopted the method of combining the improved SSA and the adaptive classifier and introduced the sine-cosine algorithm and the newly proposed labor cooperation structure. Great effect of application in the classification of lung CT images has been demonstrated. Zhang and Ding [21] designed a random configuration network based on the chaotic sparrow search algorithm, and, combined with the adaptive control factor of CSSA, it automatically updated the regularization parameters and scale factors for SCN. Thereby, the regression performance of SCN got improved when solving large-scale random configuration problems. Zhu and Yousefi [15] proposed to hold the adaptive sparrow search algorithm ASSA to optimize the seven unknown parameters of the proton exchange membrane fuel cell model in the PEMFC stack. The ultimate goal is achieving the best consistency with the empirical voltage polarization curve of the battery pack. Zhou et al. [22] successfully applied SSA to wavefront shaping and focusing by introducing a cross strategy, which solved the problem of SSA's lack of performance in high-dimensional optimization problems. Without a doubt, the improved algorithm provided a good reference for future wavefront shaping research.

Up to now, owing to the fact that the sparrow search algorithm has not been come up with for a long time, researchers are still in the exploratory stage and have not been able to develop an absolutely excellent algorithm. In order to further improve the solution accuracy and convergence efficiency of the sparrow algorithm, this paper continues to explore paths that can be improved on the basis of the predecessors and proposes the novel sparrow search algorithm called IHSSA. Improved infinite folding iterative chaotic mapping and hybrid reverse learning strategy are combined with it. The innovation points can be summarized as follows:

1. The improved infinite folding iterative chaotic map (IICMIC) is used to initialize the sparrow population. This strengthens the diversity of the initial population to a certain extent and increases the breadth of distribution.
2. A hybrid reverse learning strategy is put forward to update the position of a specific individual. Taking into account the effectiveness of reverse learning in mining new solutions, this paper uses a hybrid reverse learning strategy. After the discoverer is updated, lens reverse learning can be utilized to update the global optimal solution. After the position of the joiner is updated, the generalized opposition-based learning strategy contributes to update the current worst individual. Besides, considering the limitation of the boundary, the population can get more feasible areas as possible so as to maximize the mining.
3. The horizontal and vertical crossing strategy is introduced to update the position of the guard. The advantage of this strategy is that it can update the individual sparrows in both the horizonal and vertical angles, while maintaining the solution speed, and the range of the population can be expanded to a certain extent.

This paper follows a reasonable logical order. The first chapter introduces the research background of intelligent algorithms in recent years and some contributions made by researchers to this field. The second chapter introduces the basic sparrow search algorithm SSA. The third chapter introduces several improvement points of this paper in sequence according to the application order, shows the proposed new algorithm IHSSA, and attaches the flow chart of the new algorithm. The advantage of the algorithm is proved by time complexity analysis and Wilcoxon rank sum test, and the population distribution diagram proves its contribution to the dispersed population. In the following chapters, the new algorithm is tested on 14 standard test functions, the results are statistically tabulated, and a comparative analysis is made according to the data to verify the pros and cons of the algorithm. In Chapter 5, we apply IHSSA to a classical constraint engineering optimization problem, and the obtained data further proves the feasibility and effectiveness of the proposed algorithm. Finally, a brief summary of the work of this paper is made, and the author and his team have made some plans and prospects for the next research work.

## 2. Sparrow Search Algorithm SSA

### 2.1. Group Predation Behavior of Sparrows

In nature, as one of the common birds, sparrows live in the environment where humans live. Generally speaking, the upper body of the sparrow is brown and black, and the conical mouth is short and strong. They usually live together in groups with a clear division of labor. Some sparrows are responsible for finding food and providing foraging areas and directions for the entire population, while the remaining sparrows obtain food based on the food information the former sparrows provide. In addition, a sparrow in the population will issue an alarm in time when it realizes that danger is coming, and the entire population will quickly start backfeeding behavior.

### 2.2. SSA Algorithm Description

The proposal of SSA is based on the characteristics of sparrows' cleverness and strong memory, which well simulates the cooperative mechanism of sparrow populations in daily foraging. We will give new names to the three types of sparrows mentioned earlier. ① Those who are responsible for finding food are called discoverers. ② Those who follow the discoverers to obtain food are called joiners. ③ Some joiners will always monitor the discoverers and choose the time to compete for food resources in order to increase the rate of food acquisition. This type of joiner is called monitor. The discoverer generally accounts for 10%–20% of the entire population. The roles of the discoverer and the joiner can be exchanged, provided that the proportion relative to the entire population is constant.

The position of each sparrow is held as a solution of the algorithm. The initial positions of the sparrow represented by a matrix are as follows:

(1) $$\begin{array}{c} \left[\begin{array}{cccc} {\text{x}}_{1,1} & {\text{x}}_{1,2} & \cdots & {\text{x}}_{1,\text{d}}\\ {\text{x}}_{2,1} & {\text{x}}_{2,2} & \cdots & {\text{x}}_{2,\text{d}}\\ \vdots & \vdots & \ddots & \vdots \\ {\text{x}}_{\text{n},1} & {\text{x}}_{\text{n},2} & \cdots & {\text{x}}_{\text{n},\text{d}} \end{array}\right]. \end{array}$$

Among them, *d* represents the dimension of the problem to be optimized, and *n* represents the number of sparrow population. And then, the fitness value of all sparrows can be expressed:

(2) $$\begin{array}{c} F\left(x\right)=\left[\begin{array}{c} f\left(\left[x_{1,1\;}x_{1,2}\;\cdots \;x_{1,d}\right]\right)\\ f\left(\left[x_{2,1\;}x_{2,2}\;\cdots \;x_{2,d}\right]\right)\\ \vdots \\ f\left(\left[x_{n,1\;}x_{n,2}\;\cdots \;x_{n,d}\right]\right) \end{array}\right]. \end{array}$$

Among them, the function *f* represents the fitness function. The discoverer with better fitness will obtain food earlier in the food search process.

Since the discoverer needs to guide the foraging direction for the entire population, the discoverer can obtain a larger food search range. In the iterative process, the location of the discoverer is updated as follows:

(3) $$\begin{array}{c} X_{i,j}^{t+1}=\left\{\begin{array}{cc} X_{i,j}^{t}\cdot \text{EXP}\left(-\frac{i}{\alpha \;\cdot \text{Maxitem}}\right), & R_{2}<ST,\\ X_{i,j}^{t}+\;Q\;\cdot \;L, & R_{2}\geq ST. \end{array}\right) \end{array}$$

Among them, *X*_*i*,*j*_^*t*^ represents the current position of the *i*^th^ sparrow; *Maxitem* represents the maximum number of iterations of the algorithm; *t* is the current iteration number; *α* is a uniform number conforming to (0,1]; *Q* is a random number that obeys the standard normal distribution; *L* is a 1 *∗d* matrix with each element being 1; alarm value *R*_2_ ∈ [0,1]; safety value *ST* ∈ [0.5,  1]. Once a sparrow in the population finds a predator or other danger, an alarm signal will be issued. When the alarm value is more than safety critical value, the discoverer will lead the population to other safer areas to forage.

The formula updated position of the follower is as follows:

(4) $$\begin{array}{c} X_{i,j}^{t+1}=\left\{\begin{array}{cc} Q\cdot \text{EXP}\left(\frac{X_{\text{worst}}\;-\;X_{i,j}^{t}}{i^{2}}\right), & i>\frac{n}{2},\\ X_{b,j}^{t+1}+\left|X_{i,j}^{t}\;-\;X_{b,j}^{t+1}\right|\cdot A^{+}\cdot L, & \text{else.} \end{array}\right) \end{array}$$

Among them, *X*_worst_ represents the current global worst position; *X*_*b*,*j*_^*t*+1^ represents the global optimal value of the j^th^ dimension at the (*t*+1)^th^ iteration (that is, the best position of the discoverer); A represents a 1∗*d* matrix whose elements are randomly assigned 1 or -1, *A*^+^ Satisfy *A*^+^=*A*^*T*^(*AA*^*T*^)^−1^.

When *i* > *n*/2, it indicates that the i^th^ joiner has a low fitness level and is not able to obtain food. In order to obtain food and increase energy reserves, one must fly to other places for foraging; when *i* ≤ *n*/2, it means that the i^th^ joiner has held the best position and randomly finds a location to forage near *X*_*b*,*j*_.

The sparrows responsible for investigation generally account for 10%–20% of the total, and they always monitor and remind the entire population to take backfeeding behavior when facing danger. The position update formula of the monitors is as follows:

(5) $$\begin{array}{c} X_{i,j}^{t+1}=\left\{\begin{array}{cc} X_{i,j}^{t}+\beta \left|X_{i,j}^{t}\;-\;X_{b,j}^{t}\right|, & {\text{f}}_{i\;}\neq f_{g},\\ X_{i,j}^{t}+K\frac{X_{i,j}^{t}\;-\;X_{\text{worst},j}^{t}}{\left(f_{i}\;-\;f_{\text{worst}}\right)+\varepsilon }, & {\text{f}}_{i\;}=f_{g}. \end{array}\right) \end{array}$$

Among them, *K* is also a random number, and the range is [−1,1]; *ε* is an infinitesimal constant, and its existence avoids the situation where the denominator is 0; f_*i* _, *f*_*g*_ and *f*_worst_ represent the current fitness, the global optimal, and the global worst fitness value of the sparrow, respectively.

## 3. IHSSA

### 3.1. Infinitely Folded Iterative Chaotic Map Initialization Population

#### 3.1.1. ICMIC

The swarm intelligence algorithm needs an initialization strategy to generate an initial population and provide an initial guess for the subsequent evolution process. The difference in the initial distribution state of the sparrow population will lead the entire subsequent foraging process to the final result with a large gap. Both the convergence speed and the optimization accuracy are deeply affected. Therefore, the importance of the quality of the initial population can be realized. According to the original SSA, the population is not guided by prior knowledge; that is, it is generally randomly generated. In 1975, Li et al. proposed the concept of “chaos” for the first time in the article “Period Three Implies Chaos” and used the word chaos for the first time [23].

Considering its unpredictability, ergodicity, and parameter sensitivity, chaotic systems are special. In the field of parameter optimization, chaotic mapping can be operated to replace pseudorandom number generators in order to generate chaotic numbers between 0 and 1. Considering that chaos can only traverse all the space in a sufficient length of time, it is feasible to combine chaos into the global optimizer to improve the search performance of the latter in order to complete the optimization of the target task in a short time range [24]. Experiments have proved that the utilization of chaotic sequences for population initialization will affect the entire process of the algorithm, and better results than pseudorandom numbers can often be held. The ergodicity of chaos allows the initial state of the sparrow population to have better diversity, to avoid premature convergence, that is, to improve the global optimization accuracy and convergence, which overcomes the shortcomings of traditional optimization algorithms.

This paper applies ICMIC map, one of the most classic chaotic maps (Iterative Chaotic Map with Infinite Collapses) to initialize the sparrow population. The chaotic map was proposed in 2001 by Di He. Its basic idea is to generate a chaotic sequence in [0, 1] through the mapping relationship and then transform the chaotic sequence into the search space of the population [25]. Its higher Lyapunov exponent shows stronger chaotic characteristics than other commonly used continuous chaotic models [26]. Selecting appropriate parameters can generate a good chaotic model so as to contribute satisfactory results in practical applications. The uniform distribution test of chaotic systems by Di et al. [26] proved that the one-dimensional ICMIC presents a noise phenomenon closer to uniform distribution. Two mathematical expressions for ICMIC mapping are as follows:

Expression one:

(6) $$\begin{array}{c} x_{n+1}=\sin\left(\frac{a}{x_{n}}\right),\\ -1\leq x_{n}\leq +1,\\ x_{0}\neq 0,\\ a\in \left(0,+\infty \right),\\ \text{n }=0,1,2,\ldots . \end{array}$$

Expression two:

(7) $$\begin{array}{c} x_{n+1}=\sin\left(\frac{\alpha \pi }{x_{n}}\right)\\ \alpha \in \left(0,1\right). \end{array}$$

In expression one, *a* is a very important adjustable parameter. Experiments show that the value of *a* directly affects the mapping effect and then affects the pros and cons of the population. In the second expression, *α* also plays an important role as a control parameter.

#### 3.1.2. IICMIC

Based on the expression two in 2.1.1, this paper proposes an improved infinite fold iterative chaotic map-IICMIC. The mathematical expression is as follows:

(8) $$\begin{array}{c} x_{n+1}=\sin\left(\frac{\alpha \beta }{x_{n}}\right)\\ \beta =3\;\cos\left(r\text{and}\left(1\right)\right)+\frac{1}{2}. \end{array}$$

After a lot of experiments, it is concluded that SSA can obtain a good chaotic sequence when the value of a is in the range of (0.6, 1). Combining IICMIC with the original SSA, the initial population state generated is shown in Figure 1(a) which shows the population state distribution after initial SSA initialization, and Figure 1(b) shows the distribution of sparrow population state after initialization with IICMIC. It can be seen that the improved initialization method has greatly improved the diversity of the population, and it has greatly avoided falling into the local optimum. The value of a is set 0.9 in subsequent experiments afterwards.

In combination with SSA, we first select initial values whose number is *N* with small differences as the initial state of the population. Taking into account the parameter sensitivity of ICMIC mapping, even if the individual gap is small, it can be captured. These *N* initial values can be mapped to get the same amount of chaotic sequence and then inversely mapped to the corresponding individual search space. The initial position of the i-th individual after the change is denoted as *X*_*n*+1_^*i*^ (*i* = 1.2,…, *D*).

### 3.2. Hybrid Reverse Learning Strategy to Update the Position of the Discoverer

Opposition-based learning (OBL) is an intelligent calculation method, which is first proposed by Tizhoosh in 2005. With the in-depth research of various algorithms, OBL has been successfully applied to many intelligent algorithms [27–31]. The main idea can be summarized as follows: calculate a feasible solution and its reverse solution. Then, evaluate the pros and cons of the two, and select the required solution according to certain conditions. Research shows that the solution generated by reverse learning is better than the randomly generated solution, and the probability of reaching the optimal solution is higher. Therefore, OBL is a good method that is greatly suitable for mining new solutions in unknown fields, which increases the diversity of the population.

In the discoverer stage, a broad and flexible search mechanism is the key to guide the entire sparrow population to search for food and avoid tripping into danger. In order to better realize the lead role of discoverers, it takes researchers too much time to explore in these fields, and they put forward a series of improvement methods gradually. However, traditional learning strategies have limited ability to solve problems and can only achieve their goals in certain dimensions. In response to this problem, based on the traditional OBL, this paper proposes a hybrid reverse learning method. Not only the improved lens imaging inverse learning mechanism is applied to the update of the optimal solution in the discoverer stage, but also the generalized opposition-based learning is performed on the global worst solution. The higher optimization accuracy can be obtained in this hybrid way so as to avoid premature convergence.

#### 3.2.1. Reverse Learning Strategy Based on Improved Lens Principle to Update Optimal Position

The reverse learning strategy based on the lens principle has strong flexibility and versatility. A strong ability to explore unknown areas and dig new solutions is another advantage. The principles of this method are as follows:

Supposing that there is an object *P* with a height of *h*, and *X*_*p*_ is the projection of *P* on the *X* axis. Define *a*_*j*_ and *b*_*j*_ to be the upper and lower bounds of the solution in the j-th dimension under the current algorithm. The midpoint of the upper and lower bounds is defined as the base point *O*, and a lens with focal length *f* is placed at this point. Through the lens imaging, an image *P*′ different from *P* can be obtained. The projection of the image *P*′ on the *X* axis is denoted as *X*_*P*_′. *X*_*P*_′ is the newly generated reverse solution based on this learning strategy. The schematic diagram is shown in Figure 2.

From Figure 2, we can clearly see that *X*_*p*_ generates a new image *X*_*P*_′ under the action of the lens. According to the properties of similar triangles, we can get the following formula:

(9) $$\begin{array}{c} \frac{\left(a+b\right)/2-X_{p}}{X_{P}^{\prime }-\text{a}+b/2}=\frac{h}{h^{\prime }}. \end{array}$$

Let *h*/*h*′=*k* (k is the scale factor), and the mathematical expression of the reverse point *X*_*P*_′ can be written as

(10) $$\begin{array}{c} X_{P}^{\prime }=\frac{a+b}{2}+\frac{a+b}{2k}-\frac{X_{p}}{k}. \end{array}$$

When *k*=1, we can get

(11) $$\begin{array}{c} X_{P}^{\prime }=a+b-X_{p}. \end{array}$$

The formula above is the general form of the reverse learning strategy, and the new individuals generated by this formula are fixed. Studies have shown that, for high-dimensional complex functions, new individuals with a fixed range have a certain probability of falling into a local optimum. In the later stage of the algorithm iteration, the optimal solution generated is usually very close to the optimal solution. In order to deal with the hidden danger, we can introduce a new operator *k*^*∗*^. Changing the scale factor *k* contributes to dynamically variable and new individuals. The randomness of the solution prevents individuals from losing vitality and increases the diversity of the population. The mathematical expression of *k*^*∗*^ is as follows (the expression is implemented to the position of the i-th sparrow individual on the j-th dimension):

(12) $$\begin{array}{c} X_{P}^{\prime }=\frac{a^{j}+b^{j}}{2}+\frac{a^{j}+b^{j}}{2k^{*}}-\frac{X_{p,\text{i}}^{j}}{k^{*}}\\ k^{*}=k+\text{sin}\left(\pi \times \frac{T-t}{T}\right). \end{array}$$

Among them, *t* represents the current number of iterations, and *T* represents the maximum number of iterations.

#### 3.2.2. Generalized Reverse Learning Strategy Updates the Current Global Worst Position

With the deepening of research, more and more attempts have been made to choose the optimal solution, but the research on the current global worst position cannot be ignored. The update of the worst position can bring a better search range and make the population distribution greater. In order to maximize the diversity of individuals in the population, not only the best individuals in the discoverer stage are learned, but also the worst individuals in the sparrow group are learned in reverse strategy. Combined with the improved lens learning strategy in the previous subsection, this subsection adopts the generalized opposition-based learning (GOBL) strategy to optimize and update the current global worst position after each iteration.

The concept of generalized opposition-based learning is as follows: let the individual *x*_*i*_=(*x*_*i*,1_, *x*_*i*,2_,…, *x*_*i*,*n*_), and their dynamic search range in the j-th dimension space is [*a*_*j*_, *b*_*j*_]. *x*_*i*_′ is its reverse solution. The mathematical expression of *x*_*i*_′ is

(13) $$\begin{array}{c} x_{i}^{\prime }=k\left(a_{j}+b_{j}\right)-x_{i}. \end{array}$$

Among them, *k* is a random number that obeys a uniform distribution between (0, 1). If the value range of the reverse solution exceeds the predetermined range, the solution will be randomly generated within the dynamic search range [*a*_*j*_, *b*_*j*_] according to the following formula:

(14) $$\begin{array}{c} x_{i}^{\prime }=a_{j},b_{j}. \end{array}$$

The purpose of reverse learning is to find a new and most suitable solution. Generalized opposition-based learning (GOBL) compares the worst solution while finding it and updates the current global worst solution once. At the same time, GOBL increases the dynamic update operation of the boundary than the basic reverse learning, which means the relatively small search space. The GOBL is combined with the worst joiner update of the sparrow search algorithm. The characteristics of reverse learning are fully utilized to explore more feasible regions while improving the convergence speed of the algorithm.

### 3.3. Vertical and Horizontal Cross Strategy

The optimization speed of the SSA is very fast, and the solution accuracy is also strong. As the number of iterations increases, the sparrow population will gather around the local optimal solution to a large extent. In order to balance the global search and development capabilities of the algorithm and avoid the algorithm from falling into the local optimum, the crossover optimization algorithm is newly proposed in 2014. It is inspired by the Confucian golden section principle and the crossover operation in genetic algorithms. The experimental results demonstrate that, compared with other heuristic algorithms, the cross-optimization algorithm has excellent performance on most test functions [32].

This paper proposes to integrate the vertical and horizontal crossover strategy into the guard search stage of the sparrow search algorithm, which expands the range of the population as much as possible while preserving the speed of the solution.

#### 3.3.1. Horizontal Crossover Strategy

Horizontal crossover divides the solving space of multidimensional problem into half the population of hypercubes. In order to reduce the blind spots that cannot be reached, the horizontal crossover also searches the edge of each hypercube with a small probability. This is the guarantee that horizontal search has strong global search ability.

In this paper, two parental vigilant individuals *x*_*d*_^*t*^(*i*) and *x*_*d*_^*t*^(*j*) are crossed horizontally to generate new individuals *MSx*_*d*_^*t*^(*i*) and *MSx*_*d*_^*t*^(*j*).

(15) $$\begin{array}{c} MSx_{d}^{t}\left(i\right)=r_{1}\times x_{d}^{t}\left(i\right)+\left(1-r_{1}\right)\times x_{d}^{t}\left(j\right)+c_{1}\times x_{d}^{t}\left(i\right)-x_{d}^{t}\left(j\right), \end{array}$$

(16) $$\begin{array}{c} MSx_{d}^{t}\left(j\right)=r_{2}\times x_{d}^{t}\left(j\right)+\left(1-r_{2}\right)\times x_{d}^{t}\left(i\right)+c_{2}\times x_{d}^{t}\left(j\right)-x_{d}^{t}\left(i\right). \end{array}$$

Among them, *r*_1_ and *r*_2_ are random numbers in [0, 1] conforming to a uniform distribution, and *c*_1_ and *c*_2_ are random numbers in [−1, 1] conforming to a uniform distribution.

The offspring produced by the horizontal crossover needs to make an elite selection with their parents and retain the individuals with high adaptability. In this way, the algorithm can continuously converge to the optimal solution, which can ensure the convergence efficiency without affecting the optimization accuracy.

#### 3.3.2. Vertical Cross Strategy

The premature convergence of most swarm intelligence search algorithms is caused by a small number of stagnant population dimensions. The original purpose of introducing vertical crossover is to promote certain dimensions of the population to escape from the dimensional convergence. Differing from the horizontal crossover strategy, the vertical crossover is operated on all dimensions of the new individual. Its function is to avoid premature maturity in the later stage of SSA, which is similar to the mutation mechanism in genetic algorithm.

Assuming that there is a newborn individual *x*_*d*_^*t*^(*k*), which crosses longitudinally in the *d*_1_ and *d*_2_ dimensions, the calculation formula is as follows:

(17) $$\begin{array}{c} MSx_{d}^{t}\left(k\right)=r\times x_{d}^{t}\left(k\right)+\left(1-r\right)\times x_{d}^{t}\left(k\right). \end{array}$$

Among them, MS*x*_*d*_^*t*^(*k*) is a new individual generated after vertical crossover, *r* ∈ [0,1].

Like the individuals generated by the horizontal crossover strategy, the new individuals generated after the vertical crossover must be selected by elites with their parents. The one with high adaptability is retained as the final individual. The advantage of this is that it not only increases the possibility of seeking the best in breadth, but also chooses various dimensions and realizes the continuous improvement of the quality of the solution. Even individuals who have fallen into a local optimum have a chance to jump out.

It is not difficult to see that, after combining with the horizontal and vertical crossover, it is indeed possible to balance the exploration and mining capabilities of the algorithm to a certain extent. The bottleneck in the horizontal direction can be shifted from the vertical experiment, and the vertical gains will be immediately fed back to the horizontal cross. Then, the information will spread to the entire population. The perfect combination of the two is like a layer of mesh structure that provides maximum help for optimization.

### 3.4. Frame Work of IHSSA

In summary, in order to solve the problems of the original sparrow search algorithm, such as fast convergence speed and high accuracy, but easy to mature early, several improvement measures have been proposed. The improved ICMIC is applied in the initialization phase, and the hybrid reverse learning strategy is utilized to update the discoverer and joiner, respectively. At the same time, the vertical and horizontal crossover strategy is added in the monitor stage to realize the overall update of each stage and strive to maximize the optimization. The specific implementation steps are as follows:

**Step 1 .**

Initialize the population and its parameters, including the population size *N*, the proportion of discoverers *PD*, the proportion of guards *SD*, the dimension of the objective function set to *D*, the upper and lower bounds of the initial value set to *lb* and *ub*, the maximum number of iterations *T*, and the alarm threshold *ST*, solving accuracy *ε*.

**Step 2 .**

Employ IICMIC to initialize the population (8), generate N D-dimensional vectors Zi, and then inversely map to the corresponding individual search space. The renewal of the population ensures the diversity of the sparrow population.

**Step 3 .**

Calculate the fitness *f*_*i*_ of each sparrow, select the current optimal fitness fb and its corresponding position xb, and the current worst fitness fw and its corresponding position xw.

**Step 4 .**

According to the set ratio PD, randomly select pNum sparrows with excellent adaptability as discoverers, and the rest become joiners. Update the position of the discoverers according to formula (3).

**Step 5 .**

According to the population fitness updated by the discoverer, an improved lens-based reverse learning strategy (12) is utilized to update the optimal value.

**Step 6 .**

Update the position of the joiner according to formula (4).

**Step 7 .**

Employ the generalized opposition-based learning strategy (13) to update the current global worst value.

**Step 8 .**

Randomly generate sNum guards from the population according to the ratio SD, and perform the horizontal crossover (15) and (16) operation.

**Step 9 .**

Perform vertical crossover operation according to formula (17), compare the degree of fitness, and save the better ones.

**Step 10 .**

According to the current state of the sparrow population, update the optimal position xb, the best fitness value fb, the worst position xw, and the worst fitness value fw of the entire population during the entire foraging process.

**Step 11 .**

Determine whether the iteration is over. If the algorithm reaches the maximum number of iterations, or the solution accuracy reaches the set value, it is determined that the loop ends, and the optimization result is output. Otherwise, it returns to Step2 to continue the next iteration operation, and the current iteration number *t* satisfies *t*=*t*+1.

**Step 12 .**

Output the results of IHSSA.

The flow chart is shown in Figure 3.

## 4. Experimental Results and Analysis

### 4.1. Benchmark Function Test

In order to better verify the effectiveness of the newly improved algorithm, this paper selects 14 internationally representative benchmark functions for testing. The selected benchmark functions, which hold the function name, expression, and search interval of the function, are shown in Table 1. F1–F4 in the table are unimodal functions, usually only a global optimal value, the purpose of which is to test the local mining capability of the function. F5–F7 are multimodal functions which test the balance between exploration and mining of the function. The final selections F8–F14 are all fixed-dimensional functions. The theoretical optimal values of the 14 selected test functions are all 0.

All the algorithms mentioned are performed on Windows10 64 bit system, and the processor is Intel(R) Core(TM) i5-9300H CPU @ 2.40 GHz with 16 GB RAM. And the MATLAB R2016b simulation experiment platform is used for simulation.

### 4.2. Ablation Experiment

In order to verify the influence of the three improvement points of the algorithm on the effect of the entire experiment, an ablation experiment is hereby carried out. The comparison results are analyzed and have strong persuasion. The functions used for verification still select the 14 functions selected in the previous section, and the statistical results are divided into 5 angles according to the type and number of improvement points. These algorithms include the original SSA; the improved ICMIC initial population combined with the initial SSA is named ISSA-I; the improved algorithm combined the hybrid reverse learning strategy with the ISSA-I is named ISSA-II; the improved algorithm combined the crisscross strategy with ISSA-I is named ISSA-III; the last one is the IHSSA that combines all the innovations proposed in this paper. Integrate the data into Table 2 according to the principles above.

It can be seen from Table 2 that, in the process of improvement, the indicators of 8 functions have no obvious changes in the data. Among them, each index of the 7 functions, F1, F5, F6, F7, F9, F11, F12, and F13, reaches the optimal value of 0 in the SSA. The value obtained by the improved algorithm still keeps the optimal state. With the increase of improvement points, in the five functions of F2, F3, F4, F10, and F14, the optimization effect becomes more significant. Except for the best optimization of ISSA-III in F14, the other four functions are all the best optimization values of IHSSA and even get progress of many orders of magnitude. In F8, although there is no improvement in the two data of average and standard deviation, the optimal value has reached an improvement of 7 orders of magnitude. Overall, the IHSSA that combines all the innovation points proposed in this article has the best effect. Each innovation point has played a certain role in each step of the algorithm; especially combining IICMIC with population initialization has brought obvious results.

### 4.3. Population Diversity Analysis

Population diversity is one of the important performance indexes to measure the pros and cons of an algorithm, which can reflect whether the algorithm falls into a local optimum to a certain extent. In this paper, the population distribution map in the early stage of the iteration (the number of iterations is 10) was selected as a reference. The unimodal function F1 and multimodal function F8 proposed in the above table were selected as the research objects to show the advantages and disadvantages of IHSSA and the original SSA, as shown in Figures 4(a) and 4(b), respectively, representing the individual distribution of SSA and IHSSA on F1, and Figures 4(c) and 4(d), respectively, represent the individual distribution of SSA and IHSSA on F8. The theoretical optimal value of F1 is 0, and the theoretical optimal value for F8 is 420.

As can be seen from Figure 4, in the early stage of the algorithm iteration, the distribution in Figure 4(a) is linear, while the IHSSA in Figure 4(b) is more widely distributed. Compared with the poor aggregation state of SSA in Figure 4(c), the distribution shown in Figure 4(d) is closer to the theoretical optimal value and presents a wider distribution field. It can be seen that the improved IHSSA in this paper increases the diversity of the population to a certain extent and reduces the invalid search of individuals.

### 4.4. Comparison with Other Optimization Algorithms

14 standard test functions proposed in the previous section are utilized to test the performance of the improved IHSSA. Nine intelligent optimization algorithms, including particle swarm optimization (PSO), whale optimization algorithm (WOA), grey wolf optimization algorithm (GWO), teaching and learning algorithm (TLBO), Sparrow Search Algorithm (SSA), Chaos Sparrow Optimization Algorithm (CSSA) proposed by Lv et al. [2], LSSA improved by Zhu DL [33], GSSA improved by Chen G, and YSSA proposed by Yan et al. [34], are chosen for comparison. In order to ensure the objectivity of the experiment and the fairness of comparison, the population size and maximum iteration number of each algorithm are 100 and 500, respectively. The other parameter settings of the 8 algorithms are shown in Table 3. Considering the importance of parameter values in experimental results, the feasibility proved by a large number of experiments is the only source of value, so the data in the table are from the parameter values set by the author when each algorithm was first proposed. In order to avoid the contingency of the algorithm results, each test function is run 30 times separately. And the average value, standard deviation and optimal value of the experiment are calculated, respectively. Meanwhile, the average running time of each algorithm for optimizing in each function was recorded as a reference for improving performance. The experimental data are shown in Table 4.

It can be seen from Table 4 that, compared with the other three SSA algorithms, the same results are achieved in 7 functions; even the 6 functions F1, F5, F7, F9, F11, and F13 have found the optimal solution 0. There are obvious improvements in the remaining 7 functions, and the average value of optimization in F2, F3, and F4 has been improved by multiple orders of magnitude. Compared with the WOA, GWO, and TLBO algorithms, the optimal solution 0 is found in F5, F9, and F7, respectively, and the results in the other functions are better. Compared with the PSO algorithm, the five functions of F4, F11, F12, F13, and F14 have a significant improvement, which is particularly prominent in F4. In addition, compared with the basic SSA, the optimal values found in the three functions are improved significantly. Compared with the other two improved SSA algorithms, the results are better in the three functions of F4, F10, and F14.

In F8, apart from the GSSA, the performance of several SSA algorithms is not as good as WOA, especially in the average value. Overall, the IHSSA proposed in this paper has the best performance among the 14 functions, while the PSO has the worst performance.  Figure 5 shows the convergence curves of 8 algorithms for 10 functions. It can be seen that, among the five functions of F1, F2, F3, F6, and F12, IHSSA has the fastest convergence speed and higher convergence accuracy. In F4, F10, and F14, although IHSSA has the same convergence speed as other SSA variants, it is obviously able to obtain a better solution. For F8, WOA showed a high advantage, and GSSA shows superior optimization ability than other SSA variants. However, compared with SSA and LSSA, IHSSA performs better in convergence accuracy, but compared with GSSA, CSSA, and ISSA, the accuracy is still far from the theoretical optimal value. In terms of running time, the variant of SSA consumes more time than the original SSA. However, among several variants, LSSA and IHSSA have relatively shorter running times, and higher efficiency in the optimization process of 7 functions, respectively.

In general, IHSSA has the fastest convergence speed and better convergence accuracy; that is, the quality of the algorithm's optimal solution is better.

### 4.5. Wilcoxon Rank Sum Test

Derrac et al. proposed that, for the performance evaluation of improved intelligent optimization algorithms, data comparison only based on average, standard, and optimal values is not convincing enough. One of the necessary conditions, the quality of the statistical test results, also proves whether the algorithm has been significantly improved or not. In order to judge that the results of the improved IHSSA in this paper are significantly different from the results of other algorithms, the Wilcoxon statistical test was performed at a significance level of 5% [23]. The test principle is briefly described as follows: when *P* < 0.05, it is considered that there is a significant difference between the two algorithms. When *P* < 0.05, it indicates that the performance of the two algorithms is equivalent, and the difference is not obvious. In this article, the partial value of *P* > 0.05 is expressed as *N/A*.  Table 5 shows the *P* value calculated in the Wilcoxon rank sum test of IHSSA and other algorithms among the 14 selected benchmark functions. The results show that *P* < 0.05 accounts for the main component. The IHSSA has a greater improvement over the SSA algorithm, and its superiority is also statistically significant, which proves that the improved algorithm has a higher convergence accuracy.

### 4.6. Time Complexity Analysis

Time complexity is one of the important indicators for judging the performance of the algorithm and calculating the running cost. Analyze whether the improved IHSSA increases the time complexity from both the macro- and microperspectives. On the one hand, from a macroperspective, supposing that the maximum number of iterations of the algorithm is *M*, the dimension is *D*, and the population size is *P*, then, according to the time complexity calculation formula of the intelligent optimization algorithm, the time complexity of SSA is *O*_1_=*P* × *M* × *D*. For the improved IHSSA, although the number of cycles has been increased, the structure of the algorithm has not changed. Therefore, the time complexity *O*_2_ of the IHSSA can be calculated as *O*_2_=*P* × *M* × *D*. Obviously, *O*_1_=*O*_2_, and the time complexity has not increased in the macroscopic view. On the other hand, from a microperspective, the time complexity of IHSSA has increased to a certain extent. Assuming that the proportions of discoverers and joiners are A and B, respectively, then, the time complexity of lens-based reverse learning *O*_3_ and generalized opposition-based learning *O*_4_ is *O*_3_=*A* × *P* × *M* × *D*, *O*_4_=*M*, respectively. The increase in time complexity of the alert phase of the vertical and horizontal cross strategy update is *O*_5_=*B* × *P* × *M* × *D*. The initialization phase of IICMIC does not increase the time complexity. In summary, from a microscopic point of view, the time complexity of the improved algorithm has increased by *O*_*t*_=*O*_3_+*O*_4_+*O*_5_=(*A*+*B*) × *P* × *M* × *D*+*M*, but the increase in each step did not cause orders of magnitude. The total time complexity is still *P* × *M* × *D*.

From the above on, regardless of the macroscopic or microscopic point of view, the time complexity has not changed, which undoubtedly proves the feasibility of the algorithm improvement.

## 5. Application in Constrained Engineering Optimization Problem

### 5.1. I-Shaped Beam

The design optimization problem of I-beam is one of the classic engineering optimization problems. The goal is to minimize the vertical deflection by optimizing the width of the leg *x*_1_, the height of the waist *x*_2_ and the two thicknesses (*x*_3_, *x*_4_). The objective function and constraint conditions of this optimization problem are as follows:

Minimize:

(18) $$\begin{array}{c} f\left(x\right)=\frac{5000}{x_{3}{\left(x_{2}-2x_{4}\right)}^{3}/12+x_{1}x_{4}^{3}/6+2x_{1}x_{4}{\left(\left(x_{2}-x_{4}\right)/2\right)}^{2}}. \end{array}$$

Subject to:

(19) $$\begin{array}{c} g_{\left(x\right)}=2x_{1}x_{3}+x_{3}\left(x_{2}-2x_{4}\right)\leq 0. \end{array}$$

Variable range:

(20) $$\begin{array}{c} 10\leq x_{1}\leq 50,\\ 10\leq x_{2}\leq 80,\\ 0.9\leq x_{3}\leq 5,\\ 0.9\leq x_{4}\leq 5. \end{array}$$

### 5.2. Tree-Bar Truss Design Problem

The design problem of three-bar truss is another classic problem in engineering case studies. In order to minimize the weight constrained by stress, deflection, and buckling, it is necessary to evaluate the optimal cross-sectional area and adjust the two long rods *A*1 and *A*2 (*x*_1_, *x*_2_). The specific mathematical formulas for adjustment are as follows:

Minimize:

(21) $$\begin{array}{c} f\left(x\right)=\left(2\sqrt{2}x_{1}+x_{2}\right)\times l. \end{array}$$

Subject to:

(22) $$\begin{array}{c} g_{1}\left(x\right)=\frac{\sqrt{2}x_{1}+x_{2}}{\sqrt{2}x_{1}^{2}+x_{1}x_{2}}P-\sigma \leq 0,\\ g_{2}\left(x\right)=\frac{x_{2}}{\sqrt{2}x_{1}^{2}+x_{1}x_{2}}P-\sigma \leq 0,\\ g_{3}\left(x\right)=\frac{1}{\sqrt{2}x_{2}+x_{1}}P-\sigma \leq 0,\\ l=100cm,\\ P=\frac{2kN}{cm^{3},}\\ \sigma =\frac{2kN}{cm^{3}}. \end{array}$$

Variable range:

(23) $$\begin{array}{c} 0\leq x_{1},x_{2}\leq 1. \end{array}$$

### 5.3. Cantilever Beam

The application is a structural engineering design problem. The component part of the cantilever arm is five hollow bricks, and the purpose of the project is to increase the rigidity. Increasing the cross-sectional height of the brickwork is more conducive to improving the rigidity. If the section height increases, in order to reduce the mass or maintain the same quality, the section width must be reduced. Therefore, the size of the cross section (height or width) is the optimal parameter for this experiment. The modeling expression of this case is as follows:

Minimize:

(24) $$\begin{array}{c} f\left(x\right)=0.0624\left(x_{1}+x_{2}+x_{3}+x_{4}+x_{5}\right). \end{array}$$

Subject to:

(25) $$\begin{array}{c} g_{\left(x\right)}=\frac{61}{x_{1}^{3}}+\frac{37}{x_{2}^{3}}+\frac{19}{x_{3}^{3}}+\frac{7}{x_{4}^{3}}+\frac{1}{x_{5}^{3}}-1\leq 0. \end{array}$$

Variable range:

(26) $$\begin{array}{c} 0.01\leq x_{i}\leq 100,i=1,\ldots ,5. \end{array}$$

Three classic constrained engineering optimization problems, I-beam optimization problems, three-bar truss design problems, and cantilever beam problems, are representative in verifying the feasibility of the algorithm. The parameters and constraints of the three engineering problems are integrated in Tables 6–8, respectively. In decades of research [14, 35–41], to some extent, generations of researchers have designed many kinds of optimizers to solve these three nonlinear problems. The statistical results of these optimization methods (including the IHSSA proposed in this paper) are shown in Tables 6–8, respectively, and the optimal solutions obtained are denoted as *f*(*X*). It can be seen from Tables 7 and 8 that the IHSSA algorithm can be used in engineering optimization problems and has better performance than the original SSA algorithm. Compared with other optimizers shown in [27], the overall result is also slightly superior.

## 6. Conclusion

Based on the basic sparrow search algorithm, this paper proposes an improved sparrow search algorithm (IHSSA) that integrates infinite folding iterative chaotic mapping and hybrid reverse learning strategy so as to deal with shortcomings. Firstly, an improved infinite fold iterative chaotic map (IICMIC) is introduced in the initial population stage to increase the search range of the population. Then, in order to update the position of the global optimal value and the current worst, a hybrid reverse learning strategy is proposed to be applied after the update of the discoverer and the update of the follower, respectively. The introduction of the hybrid reverse learning strategy increases the quality of understanding and avoids falling into the global optimum. Moreover, combining the vertical and horizontal crossover strategy into the monitor stage contributes to maximizing the exploration and mining capabilities of the balance algorithm. In general, the proposal of IHSSA makes the optimization accuracy better, the development ability becomes stronger, and the algorithm's global search ability gets enhanced.

Overall, the comparison results of the solutions obtained by the 14 standard test functions also prove that the new algorithm is generally better than several well-known heuristic algorithms such as WOA, GWO, TLBO, PSO, the newly proposed SSA, and its excellent variants. IHSSA has strong stability and robustness. In terms of running time, the optimization process of the seven functions takes the least amount of time, showing high computational efficiency. In addition, the high quality of convergence accuracy is proven in the Wilcoxon rank sum test. It is proven that the update of the algorithm does not bring an order of magnitude increase in time complexity, which indicates that it is a good operation. Moreover, the application of the improved algorithm in three constrained engineering optimization problems has demonstrated its great feasibility and effect, which is better than other optimizers. This undoubtedly makes the research more meaningful. However, IHSSA research is still in its infancy.

In the follow-up research, in order to obtain better accuracy and convergence speed, we will continue to try to improve the sparrow search algorithm and other swarm intelligence algorithms. In addition, the improved algorithm and innovative points are applied to engineering optimization problems to solve practical problems, so as to broaden the application field of the algorithm and further verify the feasibility and effectiveness of the algorithm.

## Figures and Tables

**Figure 1:** Individual distribution. (a) Individual initialization map of SSA. (b) Individual distribution of IHSSA.

**Figure 2:** Lens schematic diagram.

**Figure 3:** IHSSA flow chart.

**Figure 4:** Population distribution map. (a) SSA. (b) IHSSA. (c) SSA. (d) IHSSA.

**Figure 5:** Convergence curves of eight algorithms for ten representatives test functions. *Note.* (a) corresponds to F1, (b) corresponds to F2, (c) corresponds to F3, (d) corresponds to F4, (e) corresponds to F6, (f) corresponds to F8, (g) corresponds to F9, (h) corresponds to F10, (i) corresponds to F12, and (j) corresponds to F14. The image optimization results of the four functions F5, F7, F11, and F13 have greater advantages and reach the optimal value after a short number of iterations. Since the convergence effect is too good, considering the overall beauty of the image, it will not be displayed.

**Table 1:** Fourteen benchmark test functions.

Function name	Function	Dimension	Interval
Sphere	*F*_1_(x)=∑_*i*=1_^*n*^*x*_*i*_^2^	30	[−100, 100]
Schwefel's problem 1.2	*F*_2_(*x*)=∑_*i*=1_^*n*^(Σ_*j*=1_^*i*^*x*_*j*_)^2^	30	[−100, 100]
Schwefel's problem 2.21	*F*_3_(*x*)=max_i_{|*x*_*i*_|, 1 ≤ i ≤ *n*}	30	[−100, 100]
Rosenbrock	*F*_4_(*x*)=∑_i=1_^*n*−1^[100(*x*_*i*+1_ − *x*_*i*_)^2^+(*x*_*i*_ − 1)^2^)]	30	[−30, 30]
Rastrigin	*F*_5_(*x*)=∑_i=1_^*n*^[*x*_*i*_^2^ − 10 cos(2*πx*_*i*_)+10]	30	[−5.12, 5.12]
Ackley	$F_{6}\left(x\right)=-20\text{exp}\left(-0.2\sqrt{1/n}\sum_{i=1}^{n}x_{i}^{2}\right)-\exp\left(\left(1/n\right)\sum_{\text{i}=1}^{\text{n}}\cos\left(2\pi x_{i}\right)\right)+20+e$	30	[−32, 32]
Griewank	$F_{7}\left(x\right)=1/4000\sum_{i=1}^{n}x_{i}^{2}-\prod_{i=1}^{n}\cos\left(x_{i}/\sqrt{i}\right)+1$	30	[−600, 600]
Schwefel	$F_{8}\left(x\right)=418.9829n-\sum_{i=1}^{n}x_{i}\sin\left(\sqrt{\left|x_{i}\right|}\right)$	30	[−500, 500]
Three-hump camel	*F*_9_(*x*)=2*x*_1_^2^ − 1.05*x*_1_^4^+*x*_1_^6^/6+*x*_1_*x*_2_+*x*_2_^2^	2	[−5, 5]
Colville	*F*_10_(*x*)=100*x*_1_^2^ − *x*_2_^2^+(*x*_1_ − 1)^2^+(*x*_3_ − 1)^2^+90(*x*_3_^2^ − *x*_4_)^2^+10.1((*x*_2_ − 1)^2^+(*x*_4_ − 1)^2^)+19.8(*x*_2_ − 1)(*x*_4_ − 1)	4	[−10, 10]
Bent cigar	*F*_11_(*x*)=*x*_1_^2^+10^6^∑_*i*=2_^*n*^*x*_*i*_^2^	10	[−10^10^, 10^10^]
Zakharov	*F*_12_(*x*)=∑_*i*=1_^*n*^*x*_*i*_^2^+(∑_*i*=1_^*n*^0.5*ix*_*i*_)^2^+(∑_*i*=1_^*n*^0.5*ix*_*i*_)^4^	10	[−5^10^, 10^10^]
Noncontinuous rotated Rastrigin's	*F*_13_(*x*)=∑_*i*=1_^*n*^(*z*_*i*_^2^ − 10 cos(2*πz*_*i*_)+10)+*F*_13_^*∗*^, $\hat{X}=M_{1}5.12\left(x-o\right)/100y_{i}=\left\{\begin{array}{cc} \hat{X_{i},} & if\;\left|\hat{X_{i}}\right|\leq 0.5,\\ \text{round}\left(2\hat{X_{i}}/2\right), & if\left|\hat{X_{i}}\right|>0.5, \end{array}\right)$*Z*=*M*_1_Λ^10^*M*_2_*T*_*asy*_^0.2^(*T*_*osz*_(*y*))	10	[−5^10^, 5^10^]
Levy function	*F*_14_(*x*)= sin^2^(*πω*_1_)+∑_*i*=1_^*n*−1^(*ω*_*i*_ − 1)^2^[1+10 sin^2^(*πω*_1_+1)]+(*ω*_*d*_ − 1)^2^[1+ sin^2^(2*πω*_*d*_)], Where *ω*_*i*_=1+*x*_*i*_ − 1/4	30	[−10^30^, 10^30^]

**Table 2:** Algorithm parameters

Algorithm	Parameters
GWO	*a*_*max*_=2, *a*_*min*_=0
PSO	*c*_1_=*c*_2_=1.49445
SSA	*PD* = *0.2, ST* = *0.6, SD* = 0.2
CSSA	*PD* = *0.2, ST* = *0.8, SD* = 0.2
LSSA	*PD* = *0.2, SD* = 0.2
GSSA	*PD* = *0.3, ST* = *0.6, SD* = 0.7
YSSA	*PD* = *0.2, SD* = 0.2
IHSSA	*PD* = *0.2, SD* = 0.2

**Table 3:** Ablation experiment.

Function	Index	SSA	ISSA-I	ISSA-II	ISSA-III	IHSSA
F1	Avg	0	0	0	0	0
	Std	0	0	0	0	0
	Best	0	0	0	0	0

F2	Avg	4.9592*E*-290	0	1.1301*E*-287	0	0
	Std	0	0	0	0	0
	Best	0	0	0	0	0

F3	Avg	2.9952*E*-193	1.0566*E*-230	5.119*E*-163	1*E*-233	0
	Std	0	0	0	0	0
	Best	0	0	4.7959*E*-165	0	0

F4	Avg	1.3694*E*-05	8.13949*E*-06	2.59124*E*-05	4*E*-07	2*E*-07
	Std	3.77399*E*-05	2.05064*E*-05	5.66546*E*-05	2*E*-06	8*E*-07
	Best	1.36288*E*-09	1.88962*E*-10	2.45252*E*-10	7*E*-12	0

F5	Avg	0	0	0	0	0
	Std	0	0	0	0	0
	Best	0	0	0	0	0

F6	Avg	8.88178*E*-16	8.88178*E*-16	8.88178*E*-16	9*E*-16	9*E*-16
	Std	0	0	0	0	0
	Best	8.88178*E*-16	8.88178*E*-16	8.88178*E*-16	9*E*-16	9*E*-16

F7	Avg	0	0	0	0	0
	Std	0	0	0	0	0
	Best	0	0	0	0	0

F8	Avg	3958.182107	3972.12115	2628.086289	4674.8	3377.4
	Std	712.2420957	527.205402	1002.927817	770.11	1620.5
	Best	2389.812363	3085.587428	0.014612768	3396.7	0.0008

F9	Avg	0	0	0	0	0
	Std	0	0	0	0	0
	Best	0	0	0	0	0

F10	Avg	4.82652*E*-08	3.93007*E*-08	1.53723*E*-08	6*E*-08	2*E*-08
	Std	1.02745*E*-07	8.62134*E*-08	3.49383*E*-08	2*E*-07	5*E*-08
	Best	2.87751*E*-13	2.76833*E*-14	2.82932*E*-20	2*E*-13	4*E*-15

F11	Avg	0	0	0	0	0
	Std	0	0	0	0	0
	Best	0	0	0	0	0

F12	Avg	0	0	0	1*E*-188	0
	Std	0	0	0	0	0
	Best	0	0	0	0	0

F13	Avg	0	0	0	0	0
	Std	0	0	0	0	0
	Best	0	0	0	0	0

F14	Avg	5.14521*E*-10	8.78436*E*-10	1.26547*E*-09	1*E*-11	2*E*-10
	Std	1.83095*E*-09	4.04952*E*-09	2.0902*E*-09	5*E*-11	8*E*-10
	Best	2.07524*E*-20	3.3079*E*-14	3.0117*E*-11	2*E*-15	2*E*-14

**Table 4:** Comparisons of IHSSA and other seven algorithms for 14 test functions.

Function	Algorithm	Avg	Std	Best	Run time
F1	WOA	6.47271*E*-97	2.45955*E*-96	1.4869*E*-104	0.00114
	GWO	9.58408*E*-41	1.61375*E*-40	1.85345*E*-42	0.001135
	PSO	4.51174*E*-11	6.25117*E*-11	1.31715*E*-12	0.003173933
	TLBO	2.29067*E*-85	1.79774*E*-85	2.6797*E*-86	0.0051
	SSA	0	0	0	0.001907
	CSSA	0	0	0	0.002318533
	LSSA	0	0	0	0.002167
	GSSA	3.826*E*-123	1.4763*E*-122	0	0.003030333
	YSSA	0	0	0	0.0024253
	IHSSA	0	0	0	0.00231

F2	WOA	14907.66827	7290.613484	5245.501087	0.000753
	GWO	2.01843*E*-11	4.84067*E*-11	2.37886*E*-15	0.001054
	PSO	6.159248452	3.416561147	2.274329699	0.003053
	TLBO	1.49173*E*-15	1.26326*E*-15	1.28014*E*-16	0.005033
	SSA	4.9592*E*-290	0	0	0.001873
	CSSA	0	0	0	0.001958
	LSSA	0	0	0	0.002093
	GSSA	1.03442*E*-88	1.13315*E*-87	0	0.002994
	YSSA	0	0	0	0.00206
	IHSSA	0	0	0	0.001953

F3	WOA	34.68527033	29.6668357	4.83669*E*-05	0.000001
	GWO	2.5165*E*-10	2.80518*E*-10	3.92494*E*-11	0.000071
	PSO	0.210838877	0.155290345	0.057831908	0.002197
	TLBO	2.30203*E*-34	1.48485*E*-34	3.57945*E*-35	0.004141
	SSA	2.9952*E*-193	0	0	0.000924
	CSSA	0	0	0	0.00118
	LSSA	0	0	0	0.001134
	GSSA	4.87917*E*-90	2.20121*E*-89	0	0.002007
	YSSA	0	0	0	0.001297
	IHSSA	0	0	0	0.001171

F4	WOA	28.72457614	0.198079568	27.98805166	0.000752
	GWO	1.62822*E*+35	6.51934*E*+35	38250907192	0.001087
	PSO	3.24434*E*+87	4.65939*E*+86	2.29319*E*+87	0.002976
	TLBO	420.4775663	1327.016075	21.95591078	0.004966
	SSA	1.3694*E*-05	3.77399*E*-05	1.36288*E*-09	0.001724
	CSSA	6.06157*E*-06	1.48998*E*-05	1.03023*E*-08	0.001897
	LSSA	5.93493*E*-06	1.14239*E*-05	0	0.001974
	GSSA	5.11701*E*-07	5.04167*E*-07	1.6666*E*-14	0.002881
	YSSA	1.50157*E*-05	3.02452*E*-05	2.37868*E*-09	0.002006
	IHSSA	2.40169*E*-07	8.20733*E*-07	0	0.001887

F5	WOA	0	0	0	0.000587
	GWO	1.581667461	2.939452422	0	0.001086
	PSO	45.60347387	12.12604405	24.87396229	0.003016
	TLBO	6.383023506	4.955050004	0	0.005033
	SSA	0	0	0	0.001767
	CSSA	0	0	0	0.001891
	LSSA	0	0	0	0.001917
	GSSA	0	0	0	0.0028
	YSSA	0	0	0	0.002885
	IHSSA	0	0	0	0.00188

F6	WOA	5.15143*E*-15	2.16807*E*-15	8.88178*E*-16	0.000032
	GWO	2.6823*E*-14	3.63147*E*-15	1.86517*E*-14	0.000032
	PSO	0.343589201	0.596942294	1.24699*E*-06	0.002345
	TLBO	0.031044156	0.170035847	4.44089*E*-15	0.004333
	SSA	8.88178*E*-16	0	8.88178*E*-16	0.001045
	CSSA	8.88178*E*-16	0	8.88178*E*-16	0.001243
	LSSA	8.88178*E*-16	0	8.88178*E*-16	0.001302
	GSSA	8.88178*E*-16	1.00293*E*-31	8.88178*E*-16	0.002071
	YSSA	8.88178*E*-16	1.00293*E*-31	8.88178*E*-16	0.001365
	IHSSA	8.88178*E*-16	0	8.88178*E*-16	0.001232

F7	WOA	0.00420253	0.012960719	0	0.000702
	GWO	0.001780922	0.004128695	0	0.000986
	PSO	0.017048805	0.019184635	6.22012*E*-11	0.002873
	TLBO	0	0	0	0.004866
	SSA	0	0	0	0.001613
	CSSA	0	0	0	0.001893
	LSSA	0	0	0	0.001803
	GSSA	0	0	0	0.002723
	YSSA	0	0	0	0.001993
	IHSSA	0	0	0	0.001885

F8	WOA	749.0614488	1053.51792	0.142228645	0.001887
	GWO	5984.325616	512.034691	5075.836656	0.001087
	PSO	5822.761982	781.2113436	3040.698318	0.002733
	TLBO	5050.58229	1189.147899	3306.384094	0.004777
	SSA	3958.182107	712.2420957	2389.812363	0.001487
	CSSA	1619.35044	977.2374638	217.1401425	0.001995
	LSSA	4878.962977	846.4505234	3517.371964	0.001683
	GSSA	678.1120161	1382.220669	0.000381827	0.002487
	YSSA	2178.636278	2045.618662	0.000381827	0.002057
	IHSSA	3377.438965	1620.549772	0.000815262	0.001987

F9	WOA	1.2342*E*-117	5.3288*E*-117	2.672*E*-142	0.000885
	GWO	0	0	0	0.001102
	PSO	7.15959*E*-48	2.6399*E*-47	6.0523*E*-53	0.002666
	TLBO	6.1741*E*-183	0	1.5723*E*-188	0.004666
	SSA	0	0	0	0.001424
	CSSA	0	0	0	0.001911
	LSSA	0	0	0	0.001614
	GSSA	0	0	0	0.002457
	YSSA	0	0	0	0.002011
	IHSSA	0	0	0	0.001902

F10	WOA	0.754881452	1.386931349	0.001459345	0.000757
	GWO	0.600742635	1.39373905	2.53554*E*-05	0.000965
	PSO	0.000892468	0.000922365	1.42838*E*-06	0.002883
	TLBO	3.78444*E*-06	9.24279*E*-06	3.07036*E*-08	0.004883
	SSA	4.82652*E*-08	1.02745*E*-07	2.87751*E*-13	0.001633
	CSSA	6.06071*E*-08	1.74794*E*-07	4.9792*E*-14	0.001969
	LSSA	1.87914*E*-06	3.82252*E*-06	0	0.001777
	GSSA	9.6035*E*-07	1.483*E*-06	2.07901*E*-28	0.002665
	YSSA	5.06037*E*-08	9.41366*E*-08	2.87751*E*-13	0.002075
	IHSSA	1.78222*E*-08	5.32296*E*-08	3.72464*E*-15	0.001965

F11	WOA	6.5603*E*-78	3.17192*E*-77	9.75895*E*-90	0.00132
	GWO	6.77957*E*-66	2.37196*E*-65	2.19507*E*-70	0.000106
	PSO	1.0187*E*+26	2.21398*E*+25	4.6921*E*+25	0.002255
	TLBO	4.82046*E*-85	5.52867*E*-85	1.68795*E*-86	0.004233
	SSA	0	0	0	0.000977
	CSSA	0	0	0	0.001212
	LSSA	0	0	0	0.001273
	GSSA	0	0	0	0.002087
	YSSA	0	0	0	0.001338
	IHSSA	0	0	0	0.001206

F12	WOA	6.6988*E*+16	9.54778*E*+16	39646.29751	0.000265
	GWO	2.61392*E*+15	3.73552*E*+15	1.47252*E*+14	0.000282
	PSO	2.38287*E*+43	1.23114*E*+43	4.17747*E*+42	0.002377
	TLBO	9.02546*E*+14	4.72246*E*+14	2.97075*E*+14	0.004306
	SSA	0	0	0	0.000983
	CSSA	0	0	0	0.001293
	LSSA	0	0	0	0.001166
	GSSA	0	0	0	0.001983
	YSSA	0	0	0	0.001412
	IHSSA	0	0	0	0.001282

F13	WOA	0.7	0	0	0.001367
	GWO	0.8	2.006884702	0	0.000958
	PSO	1.22453*E*+20	2.91996*E*+19	5.79476*E*+19	0.003133
	TLBO	4.87463304	0.988415075	2.761251106	0.005187
	SSA	0	0	0	0.001922
	CSSA	0	0	0	0.002064
	LSSA	0	0	0	0.002097
	GSSA	0	0	0	0.002965
	YSSA	0	0	0	0.002185
	IHSSA	0	0	0	0.002057

F14	WOA	591670353.7	3240707887	1.967264854	0.000187
	GWO	5.22374*E*+34	1.32705*E*+35	5.04003*E*+32	0.000466
	PSO	1.94575*E*+60	2.11926*E*+59	1.42718*E*+60	0.002175
	TLBO	0.320134144	0.127010931	0.093171452	0.00516
	SSA	5.14521*E*-10	1.83095*E*-09	2.07524*E*-20	0.000983
	CSSA	3.47974*E*-10	7.18343*E*-10	9.49837*E*-14	0.001377
	LSSA	1.00461*E*-06	2.21303*E*-06	1.49976*E*-32	0.001183
	GSSA	1.45943*E*-07	2.58657*E*-07	7.98889*E*-19	0.002022
	YSSA	2.20337*E*-07	6.82432*E*-07	1.49976*E*-32	0.001485
	IHSSA	1.96838*E*-10	7.70225*E*-10	2.39969*E*-14	0.001365

**Table 5:** *p* value and Wilcoxon rank.

Function	WOA	GWO1	PSO1	TLBO	SSA	CSSA	LSSA	GSSA	YSSA
F1	3.02*E*-11	3.02*E*-11	3.02*E*-11	3.02*E*-11	N/A	N/A	0.049941793	N/A	0.006518796
F2	1.21*E*-12	1.21*E*-12	1.21*E*-12	1.21*E*-12	0.333710696	N/A	N/A	4.79*E*-08	N/A
F3	1.21*E*-12	1.21*E*-12	1.21*E*-12	1.21*E*-12	0.002788006	N/A	N/A	1.93*E*-10	N/A
F4	3.02*E*-11	3.02*E*-11	3.02*E*-11	3.02*E*-11	6.53*E*-08	9.26*E*-09	0.0239	9.13*E*-04	7.49*E*-08
F5	N/A	2.15*E*-06	1.21*E*-12	1.93*E*-10	N/A	N/A	N/A	N/A	N/A
F6	2.53*E*-11	5.67*E*-13	1.21*E*-12	3.50*E*-13	N/A	N/A	N/A	N/A	N/A
F7	0.081522972	0.021577192	1.21*E*-12	N/A	N/A	N/A	N/A	N/A	N/A
F8	1.49*E*-06	5.57*E*-10	4.18*E*-09	4.12*E*-06	0.02920541	3.09*E*-06	1.61*E*-06	6.51*E*-07	0.1259
F9	1.21*E*-12	N/A	1.21*E*-12	1.21*E*-12	N/A	N/A	N/A	N/A	N/A
F10	3.02*E*-11	3.02*E*-11	3.02*E*-11	1.46*E*-10	0.222572896	0.620403721	0.003475701	0.0199	0.0271
F11	1.21*E*-12	1.21*E*-12	1.21*E*-12	1.21*E*-12	N/A	N/A	N/A	N/A	N/A
F12	1.21*E*-12	1.21*E*-12	1.21*E*-12	1.21*E*-12	N/A	N/A	N/A	N/A	N/A
F13	0.0815	0.0028	1.21*E*-12	1.21*E*-12	N/A	N/A	N/A	N/A	N/A
F14	3.02*E*-11	3.02*E*-11	3.02*E*-11	3.02*E*-11	N/A	N/A	0.049941793	N/A	0.006518796

**Table 6:** Best results for the optimal design of I-shaped beam problem.

Algorithm	Variables				Constraint		
	*x*1	*x*2	*x*3	*x*4	*g*1(*X*)	*g*2(*X*)	*f*(*X*)
IARSM	79.99	48.42	0.9	2.4	0.0869999	−1.52454	0.0131
CS	80	50	0.9	2.3216	−0.012005	−1.57002	0.01307
GWO	80	50	0.9	2.3217	−0.009059	−1.570071	0.0131
EMGO-FCR	80	50	0.9	2.32	−0.176	−1.567179	0.0131
SOS	80	50	0.9	2.3217	−0.000222	−1.570224	0.01307
AEFA-C	79.9671	49.99	0.9	2.3164	−0.560371	−1.559518	0.0131
SSA	79.99992	49.99982	0.9	2.321795732	−0.00058001	−1.570210836	0.013074174
IHSSA	80	50	0.9	2.32179226	−2.06E−08	−1.570228475	0.013074119

**Table 7:** Best results of the three-bar truss design problem.

Algorithm	Variables			Constraint		
	*x*1	*x*2	*g*1(*X*)	*g*2(*X*)	*g*3(*X*)	*f*(*X*)
GA	0.788915	0.407569	9.64*E*-07	−1.464873605	−0.53512542	263.8958857
PSO	0.788669	0.408265	4.8650*E*-07	−1.464082376	−0.535917137	263.8958434
ICA	0.788625	0.408389	8.42*E*-07	−1.463941244	−0.536057913	263.8958452
CS	0.78867	0.40902	−2.90*E*-04	−0.26853	−0.73176	263.9716
WCA	0.788651	0.408316	0.00*E*+00	−1.464024	−0.535975	263.895843
GWO	0.788648	0.408325	3.34*E*-08	−1.464014397	−0.535985569	263.8960063
ALO	0.788663	0.408283	−5.32*E*-12	−1.464062005	−0.53593799	263.8958434
MFO	0.788245	0.409467	7.71*E*-12	−1.462717072	−0.537282927	263.8959796
WSA	0.788683	0.408276	3.00*E*-10	−1.46407036	−0.53587454	263.8958434
SSA	0.788628	0.408381	5.43*E*-07	−1.463950108	−0.536049349	263.8957734
IHSSA	0.788674	0.408251	5.13*E*-09	−1.464098378	−0.535901617	263.8958427

**Table 8:** Best results of the cantilever beam design example.

Algorithm	Variables					Constraint	
	*x*1	*x*2	*x*3	*x*4	*x*5	*g*1(*X*)	*f*(*X*)
CS	6.0089	5.3049	4.5023	3.5077	2.1504	−6.45*E*-05	1.33999
MFO	5.98487	5.31672	4.49733	3.51361	2.16162	4.18*E*-09	1.33998
ALO	6.01812	5.31142	4.48836	3.49751	2.15832	−3.00*E*-06	1.33995
SOS	6.01878	5.30344	4.49587	3.49896	2.15564	1.39*E*-04	1.33996
SSA	5.99215	5.28536	4.54216468	3.482721286	2.174334383	−0.00014501	1.3401483
IHSSA	5.99349	5.33819	4.501471252	3.4892014	2.152033962	−1.92*E*-05	1.340002

## Data Availability

Some data of our team needs to be kept confidential. If necessary, please ask the corresponding author for it.
